# Spatial stimuli in films: Uncovering the relationship between cognitive emotion and perceived environmental quality

**DOI:** 10.3389/fpsyg.2022.940882

**Published:** 2022-10-17

**Authors:** Hamidreza Sakhaei, Nimish Biloria, Mehdi Azizmohammad Looha

**Affiliations:** ^1^Architectural Design, Modeling, and Fabrication Lab, Department of Architecture, Tarbiat Modares University, Tehran, Iran; ^2^Faculty of Design Architecture Building, University of Technology Sydney, Sydney, AUS, Australia; ^3^Department of Biostatistics, Faculty of Paramedical Sciences, Shahid Beheshti University of Medical Sciences, Tehran, Iran

**Keywords:** cognition and emotion, spatial stimuli, normalized place quality, psychological responses, sustainable criteria

## Abstract

**Objectives:**

The research paper establishes the impact of spatial stimulus on human cognition and emotion by studying environmental events as cues to understand how people perceive spatial qualities. The medium of film to implement visually disruptive events was used in the research to find the relationship between the subjective evaluation of space and emotional responses.

**Method:**

Ninety participants participated in watching three films showcasing unexpected spatial stimuli, thus impacting their psychological state. Standard questionnaires involving Aesthetic chills and The Self-Assessment Manikin (SAM) model were used to capture emotional responses, and Normalized Accumulated Quality (NAQ) model was used to receive space quality assessments. The Pearson correlation coefficient was subsequently used to find the association of chills and The SAM with NAQ. Univariate and multivariate regression models were also conducted to find the impact of emotional responses on NAQ.

**Results:**

A significant association of NAQ with chills (*p*-value: 0.001), pleasure (*p*-value <0.001), arousal (*p*-value: 0.016), and dominance (p-value: 0.015) was witnessed in film 1. In film 2, NAQ was significantly associated with pleasure (*p*-value <0.001), while in film 3, NAQ was highly associated with arousal (*p*-value: 0.043). According to the adjusted impact of variables on NAQ in film 1, significant impacts of chills (*p*-value: 0.028), arousal (*p*-value: 0.117), pleasure (*p*-value <0.001), and dominance (*p*-value: 0.113) on NAQ were observed. In film 2, pleasure (*p*-value <0.001) and dominance (*p*-value: 0.113) impacted NAQ using the univariate model, while only pleasure had an impact on NAQ in the multivariate model. In film 3, arousal was the only variable to impact NAQ (*p*-value: 0.043) in a univariate model. In regression analyses, higher slopes were witnessed for models in film 1.

**Conclusion:**

The experiment highlighted that using affect-based video clips can help us capture the relationship between emotional responses and perceived quality of space. The appearance of spatial stimuli can engage learning, expectation, and attention, leading to a superior improvement of cognitive ability and mental health in space. This level of understanding can help design a more sustainable place.

## Introduction

Architecture and human cognition are inseparable entities that shape the perceived quality of a designed space (Hakak et al., 2017). Understanding cognitive and psychological responses while being exposed to an architectural space can prove to be a vital area of investigation. This research accordingly focuses on studying people’s environmental perception concerning cognitively storing situation-based events, their expectation or preemption of upcoming events, the extent to which these events attract their attention, and how these events impact their emotional state. Utilizing a cinematic context has proven reliable for observing the practice of a lived space (Penz, 2017). Through a film-based space screening experiment, we can thus analyze if architectural characteristics relate to emotional changes when people observe unexpected stimuli in space. Relying on the intersection of environmental design and space cognition will contribute to sustainable criteria. The perceived surrounding built space can be addressed to highlight mental health in human-environment interactions (Liddicoat et al., 2020; Buttazzoni et al., 2021; Guzman et al., 2021).

When a person’s attention is drawn to a new environment (Sakhaei, 2020), the mind tries to contextualize it by gaining spatial understanding *via* categorizing cues (Bruner, 1973). After organizing specific space cues and ignoring the ones that disrupt perception, the mind tends to formulate a consistent projection of the perceived environment (Hakak et al., 2016). By implementing disruptive events, we can scrutinize if this consistency in projecting different environments will escalate and improve spatial cognition. In our research, we implement disruptive events as cues to elicit emotions. These unexpected events or stimuli change and deconstruct the structure of architectural elements that can plausibly impact emotions. Such events, in the conducted experiment, are formulated from spaces edited from different film spaces and aimed at stimulating the physical environment to aid observers in assessing architectural qualities. The evaluation based on film space can signify space qualities during the design process to escalate the experience of designing a more communicative and sustainable place. Thus, the related literature and theories concerning the intersection of spatial cognition, emotion, and built environments will be presented to establish their integrated role in human-environment behavior. Then, the role of the cinematic realm and film contents will be associated with the environmental perception to articulate this research’s theoretical framework.

### Cognitive emotion and environmental perception

The environment we perceive affects us at cognitive and emotional levels (Sakhaei et al., 2022). The cognitive level involves mental processing and appraisal procedures, while the emotional level refers to the adaptive reaction to the gathered information (LeDoux, 1989; Higuera-Trujillo et al., 2021). Noting that cognitive and emotional levels work interrelatedly in mind, the human-space confrontation first requires activating sensory information to exhibit cognitive behavior. A substantial literature supports the relationship between human sensory information and environmental understanding (Grodal, 2009; Schacter et al., 2011; Izard, 2013; Coëgnarts, 2017). This sensory input that facilitates the entire perception process requires the active mental reestablishment of learning, memory, expectation, and attention (Bernstein, 2018).

The human mind should thus first perform cognitive tasks during the spatial learning process to perceive and assess a spatial configuration. The Cognitive Load Theory model (Paas and van Merriënboer, 1994) depicts the impact of physical characteristics of the environment as a crucial factor in studying human behavior (Tanner, 2000, 2008). Multiple studies have highlighted the learning process as necessary in cognitive tasks (Blackwood and Muir, 1990; Li et al., 2020), with factors such as volume, density, lighting, spatial arrangement, and the presence of other people being vital physical environment characteristics to enhance learning.

### Cinematic mediation and psychological reactions

Cinema has proven itself as a practical tool to present an illusion of the apparent reality of the built environment (Smith et al., 2012). There are two critical factors in films to induce the observer’s feeling of reality: the appraisal of the film’s relative realism to personal lived experiences and the factuality or plausibility of the observed events (Rooney and Hennessy, 2013). Through film induction, creating an apparent reality can capture emotional responses (Gross and Levenson, 1995; Schaefer et al., 2010; Xu et al., 2010). The dual awareness model (Tan, 2008) brings up two different domains called Entertainment Space and Executive Space while observing film scenes. As people engage with events in films, the entertainment space tries to infiltrate the mind as if they are real, while the executive space supports the constructed imagery of the entertainment space by evaluating the plausibility and reality of the observed scene compared to the real-world environment. Meanwhile, if the observer’s attention is thoroughly drawn in by the event’s realism, their minds will perceive this as apparent reality, leading to increased emotional arousal (Rooney et al., 2012).

The Limited Capacity Model (Lang, 2000) highlights that the interaction between the medium’s content information (e.g., films), its structural information (e.g., sound effect), and the observer’s characteristics (e.g., emotional arousal) are crucial to understanding cognitive allocation in human-film interactions. Evoking cognitive abilities through realistic film events can thus help to extract space characteristics and associated emotional feedback.

### Space quality and emotional responses

The quality of architectural space substantially impacts human perception (Zawidzki, 2016a). Multiple studies show that qualities like spatial openness (Hedge, 1982; Sundstrom et al., 1982) or enclosed and open spaces (Brennan et al., 2002) relate to mental contentment. Attractive, clean, and orderly spaces can indicate a high spatial quality among students in a learning environment (Gilmore et al., 2010). Architectural theorists further suggest that complexity (implicating diversity, entropy, richness) and order are also vital structures of architectural qualities (Weber, 1995). A previous study also showed that a balanced environment escalated creativity and cognitive function (Bruer, 1997).

There are two vital factors in assessing the quality of a space: Aesthetic judgments and Emotions. These factors have illustrated an interrelationship based on the Leder model (Leder et al., 2004). Accordingly, aesthetic judgment can lead to the chills responses in art perception, first studied as strong emotional responses by Goldstein (1980). Besides, feeling chills and goosebumps have been outlined as indicators of emotional arousal in other discussions (Salimpoor et al., 2009; Laeng et al., 2016). Sadness and joy are also emotional responses studied in the context of art-elicited chills (Panksepp, 1995; Nusbaum et al., 2014). The level of arousal, pleasure, and dominance responses have been studied in a PAD model as mediating between the built environment and behavior (Mehrabian and Russell, 1974; Gifford, 2007). The valence of the stimulus signifies the engaged motivational system, while arousal illustrates the activation level during the eliciting content exposure (Bradley et al., 2001; Lang and Bradley, 2010). The dominance is the emotional power of the content or the level of feeling dominated by the emotional activation (Osgood, 1966; Lang, 1979). Consequently, the four factors of chills, pleasure, arousal, and dominance can be critical emotional responses in assessing the qualities of architectural space.

### Assessing spatial quality and emotions in the cinematic context

Selecting affect-based video content to capture the mentioned emotional responses from spatial qualities require understanding the intensity and type of affect expected from the viewer (Soleymani et al., 2009). The valence-arousal space feature is an essential factor representing the appropriate affect in film content (Hanjalic and Xu, 2005). For instance, in a hierarchical movie content analysis study, film shots were divided into calm, average, and exciting to examine valence-arousal features (Xu et al., 2008). Another study depicted a substantial increase in participants’ chills, feeling moved or touched, and goosebumps from an evoking film content (Schubert et al., 2018). Apart from emotional factors, film clips should also be controlled in terms of complexity, illumination, movements, the number of characters, and camera angle to achieve a homogenous emotional content in experiments. This control is vital since film contents can be effective in subjective assessments (Carvalho et al., 2012).

### Existing gaps and hypotheses

People react differently to their perceptions of the built environment (Küller et al., 2009). Zawidzki compiled a 20-item questionnaire to define a new subjective evaluation of a place based on normalized averaged values (Zawidzki, 2016a). Zawidzki’s study mainly focused on spatial perception and geometric properties rather than a place’s aesthetic aspects. After perusing Zawidzki’s study, we found that the interrelationship between cognitive-emotional responses and subjective evaluation of spatial qualities can shed light on human-environment behavior analyses and expand the knowledge in this research area. We referred to numerous related studies and compiled the most related papers in Table 1. This table reviews prior research that assessed cognitive and emotional responses based on different stimuli, such as using films as a mediation technique to represent the real environment to capture cognitive loads or emotional behavior. However, no similar research has discussed the related emotional responses to this definition to analyze if a space’s normalized accumulated quality correlates with or affects the normalized spatial quality assessments. Assessing the space qualities based on visual cognition can plausibly associate with the emotional states of individuals in the presence of a disruptive space-deconstructive stimulus.

**Table 1:** Related research review.

Author(s)	Discussion	Methods	Results
LeDoux (1989)	Studying interacting systems of the brain that mediate emotion and cognition	Conceptual framework reasoning	Stimulus representations, affect representations, and self-representations coincidence in working memory leads to emotional experiences
Gross and Levenson (1995)	Developing a set of films to elicit eight emotional states	Film screening assessment	Films successfully elicited amusement, anger, contentment, disgust, sadness, surprise, neutral state, and fear
Wang and Cheong (2006)	Developing a systematic approach in psychology and cinematography to address affective understanding	Extracting affective information from audio streams and films into categories	Results validate the efficacy of the audiovisual cues
Xu et al. (2008)	Analyzing films’ emotion intensity and emotion type using arousal and valence-related features hierarchically	Experimental assessments	Results show that viewers prefer to access movie content by emotion intensity levels while satisfied with the emotion detection
Dijkstra et al. (2008)	The importance of individual differences in sensitivity toward colors in healthcare environments	Stimulus screening assessments	The effects of environmental coloring on stress, arousal, and cognitive appraisal were significant from different subject scores
Schaefer et al. (2010)	Testing and developing the effectiveness of a new and comprehensive set of emotional film excerpts	Subjective assessments from the film screening	Film clips were effective in emotional discreteness, arousal, and positive and negative affect
Smith et al. (2012)	Reviewing the history of empirical investigations into movie perception from various methods	Review	Sensory-motor processing differences between movies and reality help perceive continuity in the real world
AL-Ayash et al. (2016)	Learning, physiological and emotional states can be affected by colors in private study spaces	Analysis of emotional and physiological responses	Changes in colors have a significant impact on psychophysiological properties in study environments
Hakak et al. (2016)	The role of the pre-central gyrus in perceiving abstract spatial environments	Questionnaire reports from experimental environments	Correlation between designed environments and already experienced physical world
Higuera-Trujillo et al. (2021)	Impacts of neural activity during exposure to environmental situations	Scoping review	There is great potential in the neuroarchitecture approach for future design and studies
Sakhaei et al. (2022)	Examining if film stimuli help perceive architectural qualities to highlight mental health and improved cognitive tasks	Psychophysiological assessments	The intensive disruption of architectural elements indicates improved cognitive perception of spatial qualities, and enhanced interaction and can signify sustainable design criteria

In this research, we hypothesize that by ignoring unexpected events *via* the mediation of cinematic spaces, the mind would enhance its perception of the observed environment and improve mental health by assessing the quality of architectural space. We will also analyze if space-related events can change participants’ emotional states. Additionally, we will scrutinize which psychological and emotional factors relate to or affect the quality and characteristics of space.

## Materials and methods

### Study population and sampling method

We selected 90 participants (half male, mean age 26, SD 2.69) of Iranian ethnicity who were university students or employees. The chosen demographic belonged to an age group of 20–30 to capture homogenous behavioral feedback from the experiment. This demographic control is primarily due to possible human personality changes (like past experiences) that can affect assessments of different age groups (Khaleghimoghaddam and Bala, 2018). Regarding the films’ selection, we ensured that no individual had any experience of watching any of the movies previously to create a sense of novelty as regards space-related assessments. The participants were briefed regarding the procedural aspects of the experiment before the test began. This briefing included adequate resting time for each participant and having a meal before the experiment began. All of the participants reported as healthy with no mental or physical difficulty. Participants were also asked to avoid smoking, drinking alcohol, or caffeine at least 4 h before the test to avoid over-stimulation. The experiment protocol was validated and conducted under the ethical standards laid down in the 1964 Declaration of Helsinki and its later amendments or comparable ethical standards.

### Editing film sequences

Three film clips from cinematic movies were edited in a shorter format for this experiment based on two criteria. The first criterion for selecting the films was *space narration*, implying that the screened space in each clip and the depicted architectural elements therein would potentially influence the observers’ attention irrespective of the film’s script. The second criterion involved the presence of a *disruptive and evoking event* in all three film spaces such that the architectural elements therein were deconstructed. By weakening the influence of the script per clip (to avoid critical storyline and dialogs), the architecture of featured spaces within the clips was prioritized to influence the audience’s perception.

To fulfill these two criteria, we focused on particular scenes in which a one-point perspective and point-of-view or eye-level-view shots were featured in the clips. Accordingly, the film form analysis system (Bordwell et al., 1993) was regarded as a reference to extract standard scenes to depict the best affective experience of observing film spaces and space configurations. This camera height and angle choice could help our depicted spaces impart an illusion of being present within the visualized spaces. Face validity of the film clips’ final editing was examined by sending the final films to experts and academics in the fields of architecture and cinema to identify problems with the clarity of film contents to appropriately deliver the architectural space qualities based on our criteria. The video contents were then revisited and finalized based on experts’ feedback.

Thus, three film clips with an average of 5 min duration and a total of 15 min were edited for the experiment. The first and last 2 min of each film narrate a classic cozy home space, while the middle one and a half minutes show evoking events that change the physical shape of architectural elements. The house space was chosen to arouse a sense of familiarity within the participants.

Each clip is split into three parts; the ordinary scene in the first part shown to subjects allows them to be immersed in the space, thus allowing them to get acquainted with spatial characteristics. The middle section illustrates the event scene in which the previously shown architectural elements get destroyed and lose their function. In the third or final part of each movie following the event scene, subjects watched the same first part of the clip (Figure 1). They watched the repeated scene so that we could assess their cognitive responses and emotions that could have been possibly affected by the middle scene’s disruptive events. Participants’ perception of spatial quality and emotions were assessed by conducting three questionnaires-based surveys during the screenings.

**Figure 1:** Research design.

### Film plot summaries and details

Table 2 describes plot summaries and scenes’ details of the three films.

**Table 2:** Plot summaries and space-related features in the film clips.

Film name	Plot summary	Pre-event scene details	Event scene details
Film 1: *The Money Pit (1986)*	A young couple pays a visit to a classic architecture house to buy the place. As the house needs renovation to satisfy their desires, however, unpredictable accidents devastate the couple’s renovation process	The young couple checks the house to conclude if it is proper to buy. They start the renovation together to make it suitable to live for their future	The front door falls during the renovation, and the interior main stairs collapse. The electrical wiring in the kitchen catches fire while the tiles shatter. The chimney in the bedroom gets demolished when they lit the fire
Film 2: *Zathura: A Space Adventure (2005)*	Two young kids live with their father. As soon as their father leaves the house for a business, the lonely kids face strange events inside the house while playing a board game	An ordinary father-son play inside the house depicts a happy weekend in a family. The kids use the living room, stairs, and kitchen as playgrounds	The house gets hit by multiple fireballs that pierced the roof, the interior walls, and the ceiling and frightened the children. The kids run away for shelter as they watch their house gets demolished
Film 3: *I, Robot (2004)*	Robots will work as human servants in the future. While there are strict rules to control them, a detective has to determine if a robot has violated the regulations and murdered a person	The detective walks into a vacant house for investigation. He suspiciously walks into the corridor, uses the stairs, and searches the private room for clues. At least for a while, he finds no unusual activity	A giant robot starts to invade the house from the outside. It destroys the walls and continues the demolishment until the place turns to ashes. The detective runs away to save his life during the invasion

### Data collection of biofeedback and psychological measurements

We tried to conduct the research in the same timeline every day to create a more homogenous psychological atmosphere for participants. The experiment was performed between 11 a.m. and 2 p.m. in the same room with a constant temperature of 25 degrees Celsius for all subjects. We chose this timeline as people’s consciousness level could be appropriate enough to observe the films and evaluate the spaces. We tried to perform data collection in a single season of the year to preserve the homogeneous mental situation of participants that could be related to weather conditions. Accordingly, the tests were performed from September to December, which is the Autumn season in the experiment’s location.

Three standard questionnaire-based surveys were conducted to capture psychological changes during the film screenings. Questionnaires including Aesthetic Chills, The Self-assessment Manikin, and Normalized Accumulated Quality were filled out in paper and pencil format to assess emotional responses. The Aesthetic Chills (chills) questionnaire consisted of 10 questions about emotional reactions from the films’ observations. According to Silvia and Nusbaum (2011), the chills test could serve as a standard assessment test wherein people engage with art forms such as movie content. Participants can also write down in detail their self-description of emotional state for each questionnaire’s item. The Self-Assessment Manikin test (SAM) involved gathering information pertaining to the participant’s feelings of pleasure, arousal, and dominance using a 9-point scale. The SAM test describes individuals’ emotional feelings regarding three independent characteristics: pleasure, arousal, and dominance (Bradley and Lang, 1994). In this model, pleasure represents a continuous feeling ranging from severe sadness to extreme joy when watching different film sequences. Arousal illustrates the mental activity ranging from feeling asleep to an unpleasant thrill. Dominance is related to the sense of being controlled and limited when exposed to various events in the movies (Mehrabian and Russell, 1974). The Normalized Accumulated Quality (NAQ) involves a human subjective evaluation of geometrical characteristics in space (Zawidzki, 2016a). The NAQ is focused on assessing spatial perception as opposed to aesthetic features of a space.

After letting the participants feel relaxed and calm in the room where the experiment was conducted, the participants were briefed regarding the experiment procedure. The candidates were specifically instructed to assess the observed architectural details and spatial features thoroughly. The participants sat in front of a 15-inch laptop with loudspeaker audio to view the movie contents. After they watched the ordinary sequence, we paused the clip and asked them to fill out the chills, SAM, and NAQ questionnaires related to the first 2-min scene. Upon completing the three questionnaires, we continued screening the second scene with disruptive events alongside the ordinary scene without a pause in between. This was followed by the ordinary scene that was precisely the one screened in the first part of the movie. The film clip was not paused while transitioning from the second scene to the third scene, thus allowing the participants to assess the ordinary space based on the psychological changes that affected their emotions in the middle of the movie. Post this exposure, the participants were asked to complete the same chills, SAM, and NAQ survey again; Data was thus gathered for two distinct phases: pre-event and post-event, with two entirely identical scenes (scenes 1 and 3) with the latter one hypothesized to have been impacted by cognitive stimuli. This protocol was executed for all films. The participants were separated into three groups of thirty people per group for each movie. Additionally, we captured a video from each subject during their film screenings to report an observational analysis of apparent psychophysiological changes.

### Statistical analyses

The Pearson correlation coefficient was performed to evaluate the association between NAQ and variables including chills, pleasure, arousal, and dominance in different films. The impact of chills, pleasure, arousal, and dominance on NAQ was evaluated using the univariate regression model. The adjusted impact of variables on NAQ was assessed using a multivariate regression model by different films, meaning that the adjusted impacts of chills, pleasure, arousal, and dominance on NAQ were compared between the three films. R-squared was reported to measure the proportion of the variance for a NAQ explained by an independent variable. The variance inflammatory factor (VIF) was used as an indicator of multicollinearity, which is a statistical concept where several independent variables in a model are correlated. Two variables are assumed to be significantly collinear if their correlation coefficient is ±1.0. All analyses were conducted using R (version 4.0.2) and SPSS (version 26). *p*-values <0.05 were regarded as statistically significant.

## Results

Analyzing the NAQ components resulted in identifying that the ‘Harsh’ factor showed the highest fluctuation between pre-event and post-event evaluations (−3.00 for Film 1, −3.10 for Film 2, and −3.60 for Film 3). The ‘Chaotic’ (−2.80 for Film 1, −2.80 for Film 2, and −3.10 for Film 3) and ‘Artificial’ (−1.80 for Film 1, −1.30 for Film 2, and −3.00 for Film 3) factors also had the highest negative impacts on assessing of space qualities. Events had the most positive impact on the Diverse factor of NAQ (−0.50 for Film 1, +0.90 for Film 2, and +0.50 for Film 3). Overall, the Film 3 event had the highest impact on understanding the NAQ among the three film spaces.

The association between NAQ and variables such as chills, pleasure, arousal, and dominance are reported in Table 3. In film 1, NAQ was significantly associated with chills (0.56; 95% CI: 0.25, 0.76), pleasure (0.87; 95% CI: 0.73, 0.93), arousal (0.4; 95% CI: 0.08, 0.69), and dominance (0.44; 95% CI: 0.09, 0.69). This report illustrates that participants’ emotional states were significantly related to understanding the quality of space. The disruptive events in film 1 led to a substantial difference in evaluating normalized spatial qualities between pre-event and post-event scenes and highlighted a meaningful relationship with emotional feelings. There was also a significant positive relationship between NAQ and pleasure (0.72; 95% CI: 0.47, 0.85) in film 2. In film 3, however, the correlation between NAQ and arousal was observed to be positive and significant (0.37; 95% CI: 0.01, 0.64). The overall association of emotional feelings with normalized space quality depicts that the subjective assessments of space qualities could significantly impact the level of feeling pleasure and arousal. In some scenes, the high correlations of chills and dominance with assessing the space quality were observed.

**Table 3:** The association between NAQ score and variables including chills, pleasure, arousal, and dominance.

Film name	Variables	Pearson correlation (95% CI)	Value of *p*
1	NAQ – Chills	0.56 (0.25, 0.76)	0.001
	NAQ – Pleasure	0.87 (0.73, 0.93)	<0.001
	NAQ – Arousal	0.44 (0.08, 0.69)	0.016
	NAQ – Dominance	0.44 (0.09, 0.69)	0.015
2	NAQ – Chills	0.26 (−0.11, 0.57)	0.164
	NAQ – Pleasure	0.72 (0.47, 0.85)	<0.001
	NAQ – Arousal	−0.12 (−0.46, 0.26)	0.541
	NAQ – Dominance	0.36 (−0.01, 0.64)	0.050
3	NAQ – Chills	0.17 (−0.20, 0.50)	0.362
	NAQ – Pleasure	0.18 (−0.20, 0.50)	0.354
	NAQ – Arousal	0.37 (0.01, 0.64)	0.043
	NAQ – Dominance	0.32 (−0.05, 0.61)	0.087

The 95% CI was calculated for bivariate correlation variables considering the bias adjustment.

Table 4 shows the crude and adjusted impact of variables on the NAQ across different films. According to the results of film 1, the average NAQ was raised for each unit increase in the chills (0.73; 95% CI: 0.32, 1.4), dominance (0.17; 95% CI: 0.04, 0.31), arousal (0.20; 95% CI: 0.04, 0.36) and pleasure (0.28; 95% CI: 0.22, 0.35) factors. A significant impact was also found on NAQ for adjusted chills (0.37; 95% CI: 0.04, 0.70) and pleasure (0.31; 95% CI: 0.23, 0.39) factors. Accordingly, the emotional changes in participants illustrated a reasonable trend with changes in perception of spatial qualities. Subjects’ emotional changes from film 1’s space-related stimuli illustrated an impact on architectural quality assessments when we adjusted the impact of each variable on normalized space quality. In film 2, the significant impact of dominance (0.13; 95% CI: 0.00, 0.26) and pleasure (0.23; 95% CI: 0.14, 0.32) factors on NAQ was observed using the univariate model, whereas only the adjusted effect of pleasure factor on NAQ remained significant throughout the multivariate model (0.23; 95% CI: 0.15, 0.31). This report shows that feeling dominated and pleased among emotional responses in film 2 could influence normalized space quality judgments more than chills and arousal. According to film 3 and the univariate model, arousal was the only variable that significantly impacted the NAQ (0.12; 95% CI: 0.00, 0.23). The adjusted R-squared for films 1, 2, and 3 was 0.78, 0.59, and 0.05, respectively. VIFs were <5 for all variables. As shown in Figure 2, the linear regression was fitted for NAQ and other variables. Higher slopes were illustrated for models in film 1, showing a more significant impact of emotional responses on perceiving normalized space quality than events in films 2 and 3.

**Table 4:** The crude and adjusted impact of dominance, arousal, and pleasure on the NAQ by film name.

Film name	Variables	Univariate regression			Multivariate regression			
		Coefficient (95% CI)	Value of *p*	*R*^2^	Coefficient (95% CI)	Value of *p*	Adjusted *R*^2^	VIF
1	Chills	0.73 (0.32, 1.4)	**0.001**	0.32	0.37 (0.04, 0.70)	0.028	0.78	2.03
	Dominance	0.17 (0.04, 0.31)	**0.015**	0.20	−0.08 (−0.18, 0.02)	0.113		1.93
	Arousal	0.20 (0.04, 0.36)	**0.016**	0.19	−0.09 (−0.21, 0.03)	0.117		2.13
	Pleasure	0.28 (0.22, 0.35)	**<0.001**	0.75	0.31 (0.23, 0.39)	<0.001		1.93
2	Chills	0.28 (−0.12, 0.67)	0.164	0.07	0.19 (−0.13, 0.51)	0.236	0.59	1.55
	Dominance	0.13 (0.00, 0.26)	**0.050**	0.13	0.09 (−0.02, 0.20)	0.113		1.52
	Arousal	−0.06 (−0.27, 0.14)	0.541	0.12	−0.01 (−0.15, 0.13)	0.883		1.14
	Pleasure	0.23 (0.14, 0.32)	**<0.001**	0.51	0.23 (0.15, 0.31)	<0.001		1.08
3	Chills	0.12 (−0.14, 0.378)	0.362	0.03	0.06 (−0.36, 0.47)	0.789	0.05	2.75
	Dominance	0.12 (−0.02, 0.26)	0.087	0.10	0.09 (−0.11, 0.29)	0.371		2.10
	Arousal	0.12 (0.00, 0.23)	**0.043**	0.14	0.05 (−0.18, 0.28)	0.662		4.04
	Pleasure	0.09 (−0.11, 0.29)	0.354	0.03	0.09 (−0.14, 0.32)	0.418		1.40

NAQ is the dependent variable; VIF, Variance Inflammatory Factor. Bold values show that they are significant.

**Figure 2:** Scatter plot showcasing the arousal, chills, dominance, and pleasure variables as the predictors of NAQ.

## Discussion

This research tried to understand the impact of emotion-eliciting stimuli in space on environmental perception. Since environmental quality is beneficial to achieving a sustainable and communicative design (Li et al., 2021), we relied on human subjective evaluation (HSE) of space, previously developed by Zawidzki (2016b), to capture the association of normalized factors of spatial quality with chills, pleasure, arousal, and dominance in three films. Besides this, significant psychological feedback was also extracted by editing affect-based video clips with a potential valence-arousal feature (Soleymani et al., 2009). Based on previous experiments by Xu et al. that categorized a film’s content into calm, average, and exciting (Xu et al., 2008), we divided our scenes into pre-event, event, and post-event in order to systematically compile the feedback from the participants. We also standardized the camera angle, movements, and other space-related factors to control the experiment, as mentioned in an earlier study (Carvalho et al., 2012).

Our assessment revealed that the participants’ expectations changed from the pre-event scenario where they tried to memorize the environment to the event scene. It was also observed that during the event scene, participants’ attention to architectural qualities had been substantially elevated and hence, impacted their post-event responses. This could have also impacted the assignment of a superior form of attention to the disruptive events when they scored the post-event scene’s assessments. As previously validated by Bernstein (2018), this process can highlight the critical role of sensory information in determining cognitive behavior (Smith et al., 2012). During the event scene, significant alterations to the physical environments occurred in spatial arrangements, lighting, and the forms of architectural elements. While changes in the physical environment’s elements improved the overall spatial perception of participants, the experiment can validate the Cognitive Load Theory, which discussed the impact of spatial characteristics on environmental learning improvement. As discussed in the literature, order, diversity, and a balanced environment influence the perception of space and cognitive function. Likewise, after participants’ subjective evaluation of space in the three films, NAQ’s negative factors of Harsh, Chaotic, and Artificial were the most influential items impacted by post-event evaluation. On the contrary, the positive factor of “Diverse” was the most noticeable item affected by the events.

In the experiment, almost all emotional responses correlated significantly with the subjective evaluation of space. Among chills and PAD variables, both pleasure and arousal highlighted their substantial association with the evaluation of space. Similar studies also validated that utilizing film content stimuli elicited emotional feelings in participants (Gross and Levenson, 1995; Schaefer et al., 2010). Higher correlation and impact of emotional arousal with space quality assessments indicate that the spatial stimuli could possibly represent categorized cues (Bruner, 1973). Subjects’ broader attention to architectural details may illustrate the role of spatial stimuli in creating a transcendent projection of the environment compared to the normal situation. The emotional arousal can indicate that the events in the films might have helped establish an apparent reality by shifting from entertainment space to executive space discussed in Dual Awareness Theory (Tan, 2008). Participants’ engagement with the movie contents alongside emotional behavior elevated after the event scene, indicating their strong interaction with the scenes’ content and structural information as explained in the Limited Capacity Model. In Lang’s LCM model (Lang, 2000), changes in space structure and the deconstruction of elements are integrated with the viewer’s emotional states. As a result, we tried to focus on mental and cognitive aspects of space to demonstrate the importance of enhanced perception in sustainable design thinking.

The high association of chills and arousal with NAQ may also show that our experiment may explain the interrelationship between aesthetic judgments and emotion in space evaluation mentioned in the Leder model (Leder et al., 2004). Accordingly, the art-eliciting judgments in our experiment were followed by chills and goosebumps (Salimpoor et al., 2009; Laeng et al., 2016), feeling joy (Panksepp, 1995; Nusbaum et al., 2014), and PAD (Mehrabian and Russell, 1974; Gifford, 2007). The highest slopes of regression graphs were reported for the impact of chills and PAD on NAQ in film 1. The factors of chills and PAD as predictors for NAQ also showed high slopes for films two and three, demonstrating a meaningful relationship with NAQ. To validate the psychological reports of participants from observational data collection, we relied on the video-recorded data from their apparent psychophysiological changes and discovered minor alterations in pupils’ size, skin tone color, and even slight goosebumps during the event scenes. In addition, some individuals reported being aroused and overwhelmed by the space stimuli. Conversely, subjects reported being more relaxed with no apparent arousal in their body or face during the pre-event scenes. This observational study can demonstrate a sufficient alignment between psychophysiological responses and observational analyses.

According to our results, the adjusted impact of chills and PAD variables on the space quality assessments depicted a meaningful increasing trend as the average NAQ increased with elevated emotional arousal. However, among the three films, film 1’s post-event evaluation signified a stronger relationship between emotional responses and NAQ assessments both in correlation and regression analyses. In film three analyses, the arousal factor was mainly associated with the NAQ compared to other variables, meaning that the events of film three highly intensified the level of arousal than in the other two films. It can be construed that the structure of the events in film 1 was more indicative of apparent reality than in the other films. In film 1, real architecture elements shatter without significant visual effects. In the second and third films, subjects witness the same deconstruction of architectural elements but with moderate visual effects that intensify the events. The lower association of emotional responses during spatial assessments in films 2 and 3 may prove that the higher level of assuming the environment as an Entertainment Space can impact the judgment of spatial character. As mentioned in the dual awareness theory (Tan, 2008), in the second and third films, the lower level of engagement with events led to perceiving the environment only as an entertainment space. In contrast, film 1’s events could possibly lead the Executive Space to support the constructed imagery of the Entertainment Space by creating a higher association of emotional responses with the perception of spatial qualities. Capturing the association between psychological aspects of space and environmental qualities helped us notice the interrelation between sustainable design thinking and environmental research.

The overall association of chill and PAD with subjective evaluation of space demonstrated that normalized accumulated quality could be related to emotional states of feeling goosebumps, enjoyment or sadness, aroused, and dominated. We tried to establish a standard and controlled experiment to simulate real physical environments through the mediation of film context to capture the association between normalized space quality perception and emotional arousal. This mediation of cinematic context can help us understand how the human mind learns, memorizes, and judges its surroundings. Hence, we will be able to improve our built environment by enhancing spatial cognition and environmental interactions. This improvement can validate more sustainable and communicative space criteria in an interactive environment by influencing designers to highly regard cognitive emotions and space qualities within the communication discussion.

## Conclusion

This study highlighted that using affect-based video clips focusing on space-related stimuli can be an operational approach to capture the association of psychological responses with the perceived quality of a normalized place. By introducing spatial stimuli in a conventional spatial environment, the mind’s cognitive ability can be enhanced by improving the learning process and categorizing events as cues to improve environmental perception. The impact of events on emotional changes can help understand the intensity of cognitive load to assess spatial qualities. Capturing the psychological states of individuals and their relationship with spatial judgments, especially when people are exposed to environmental stimuli, can contribute to designing a highly sustainable place.

## Limitations and future research

In this study, we focused on the affective responses from different groups of participants from the same culture. However, the affective responses can vary from person to person and culture to culture. An affect representation of particular individuals could be controversial and generalized to a broad population (Wang and Cheong, 2006). We propose that this study be conducted for a broader group of people with different nationalities or experiences to consider people’s preferences and variety, thus promoting efficient affect analyses of space stimuli. Another important matter that requires critical attention for future research is controlling the film content parameters. Accordingly, the environmental stimulation in films may differ from the real environment and lead to the result distortions. This important criterion should be highly noted when the self-evaluations are prone to bias since they mainly assess the conscious human responses to the space (Schwarz and Strack, 1999). We suggest that future similar studies reflect the possible unconscious aspects when measuring individuals’ cognitive activities in mediated environments like films by noting that most emotional states appear at the unconscious level (Zaltman, 2003).

## Data availability statement

The original contributions presented in the study are included in the article/supplementary files, further inquiries can be directed to the corresponding author.

## Ethics statement

The studies involving human participants were reviewed and approved by Department of Physiology, Tarbiat Modares University. Written informed consent for participation was not required for this study in accordance with the national legislation and the institutional requirements.

## Author contributions

HS and NB: conceptualization, methodology, software, visualization, funding acquisition, investigation, review, editing, validation, project administration, and supervision. HS and ML writing original draft, data curation, and formal analysis. All authors contributed to the article and approved the submitted version.

## Conflict of interest

The authors declare that the research was conducted in the absence of any commercial or financial relationships that could be construed as a potential conflict of interest.

## Publisher’s note

All claims expressed in this article are solely those of the authors and do not necessarily represent those of their affiliated organizations, or those of the publisher, the editors and the reviewers. Any product that may be evaluated in this article, or claim that may be made by its manufacturer, is not guaranteed or endorsed by the publisher.
